The article "Speech as a Biomarker for COVID-19 Detection Using Machine Learning" was published in 2022. Journal: Comput Intell Neurosci.

# Speech as a Biomarker for COVID-19 Detection Using Machine Learning

**DOI:** 10.1155/2022/6093613

**Published:** 2022-04-18

**Authors:** Mohammed Usman, Vinit Kumar Gunjan, Mohd Wajid, Mohammed Zubair, Kazy Noor-e-alam Siddiquee

**Affiliations:** ^1^Department of Electrical Engineering, King Khalid University, Abha 61411, Saudi Arabia; ^2^Department of Computer Science and Engineering, CMR Institute of Technology, Hyderabad, India; ^3^Department of Electronics Engineering, ZHCET, Aligarh Muslim University, Aligarh 202002, India; ^4^Department of Computer Science and Engineering, University of Science and Technology, Chittagong, Bangladesh

## Abstract

The use of speech as a biomedical signal for diagnosing COVID-19 is investigated using statistical analysis of speech spectral features and classification algorithms based on machine learning. It is established that spectral features of speech, obtained by computing the short-time Fourier Transform (STFT), get altered in a statistical sense as a result of physiological changes. These spectral features are then used as input features to machine learning-based classification algorithms to classify them as coming from a COVID-19 positive individual or not. Speech samples from healthy as well as “asymptomatic” COVID-19 positive individuals have been used in this study. It is shown that the RMS error of statistical distribution fitting is higher in the case of speech samples of COVID-19 positive speech samples as compared to the speech samples of healthy individuals. Five state-of-the-art machine learning classification algorithms have also been analyzed, and the performance evaluation metrics of these algorithms are also presented. The tuning of machine learning model parameters is done so as to minimize the misclassification of COVID-19 positive individuals as being COVID-19 negative since the cost associated with this misclassification is higher than the opposite misclassification. The best performance in terms of the “recall” metric is observed for the Decision Forest algorithm which gives a recall value of 0.7892.

## 1. Introduction

The most basic functions of the human body are usually monitored by measuring the vital signs—temperature, heart (pulse) rate, respiratory (breathing rate), and blood pressure [1]. These are usually measured using medical devices, but nowadays, easy to use and low-cost devices and smart gadgets are available which allow measuring temperature, pulse rate, and blood pressure at home, even by nonmedical professionals. Various types of sensors, present in such devices, sense some signal generated by the human body, process the signal, and provide a reading of the vital sign in a simple and easy to interpret format. It is therefore necessary to connect the devices/sensors at appropriate points on the human body to obtain the desired measurements. The placement of such sensors on the body is invasive and intrusive and causes inconvenience to the patient/individual. This is particularly true when monitoring professional athletes and sports persons while they are performing intense exercise/training. Moreover, it does not allow measurement of body parameters without attaching the device/its sensors (probes) to the body or from a remote location; i.e., the patient has to be at the same location as the medical device. This article investigates the use of speech as a biomedical signal to detect COVID-19 based on a statistical analysis of speech and binary classification using machine learning. Speech characteristics of an individual get altered as a result of physiological and emotional changes [2–6]. Other factors that can cause physiological changes in the body are changes in health conditions, aging, stress, pollution exposure, and physical activity. There is significant evidence from the literature that clearly establishes a correlation between the characteristics of human speech and the physiological parameters of the speaker. A correlation between heart-related parameters such as heart rate, electrocardiogram (ECG) features, and the influence of heart function on speech characteristics has been shown in [7–13]. In [14], the variation of speech characteristics due to physical activity is demonstrated, and the effect of physical activity and fitness level on heart rate is shown in [15]. Physiological changes due to physical activity also depend on the regularity, duration, and intensity of the activity performed [16]. A correlation between speech and blood pressure is established in [17], and a method to detect emotions from speech is described in [15]. It is also established in the literature that tiredness can also affect an individual's speech and can cause speech to become slurred (dysarthria) [18]. Noncontact methods to measure physiological parameters based on image and video processing have also been investigated and reported in the literature [19,20]. Noncontact methods based on speech, images, and video can facilitate remote monitoring, telemedicine, and smart healthcare which are expected to play a major role in future healthcare infrastructures.

The article "Speech as a Biomarker for COVID-19 Detection Using Machine Learning" was published in 2022. Journal: Comput Intell Neurosci.

The COVID-19 pandemic era has necessitated and triggered an enormous amount of research into such noncontact-based diagnostic methods to detect COVID-19 using machine learning and deep learning [21–30]. A review of COVID-19 diagnostic methods along with prevention tools and policy decisions for COVID-19 management is provided in [31]. Artificial intelligence-based COVID-19 diagnosis tools are not without pitfalls. A critique of AI-based tools being given emergency authorization by regulatory bodies indicates that many such tools have been developed using small or low-quality datasets [32], concluding that AI could be useful in dealing with the COVID-19 pandemic but requires more detailed investigation and validation. Several research studies based on artificial intelligence are ongoing not only to detect COVID-19 but also to predict and understand the effects of the pandemic and be prepared for eventualities. A method to detect COVID-19 using machine learning on symptoms is proposed in [33]. COVID-19 detection based on the application of AI on X-ray and computerized tomography (CT) images is reported in [34–41]. In [42–44], detection of COVID-19 by applying machine learning to routine blood examination data has also been reported. AI-based systems to predict the deterioration of COVID-19 patients toward severe disease have been presented in [45–47], and prediction of mortality risk among COVID-19 infected individuals using AI is also available in the literature [48–50]. The COVID-19 pandemic has indeed necessitated and highlighted the need for interdisciplinary and transdisciplinary approaches to diagnose, treat, and manage not just COVID-19 patients but also to address medical problems in general [51]. The challenges involved in the use of AI for COVID-19 are elaborated in [52]. Several research groups [53–56] are actively investigating the use of speech sounds, cough sounds, and breathing/respiratory sounds to detect COVID-19 by analyzing these sounds using artificial intelligence algorithms.

## 2. Materials and Methods

### 2.1. Data Used in This Study

Speech recordings used in this study comprise two categories—speech from healthy individuals with no known preexisting medical conditions at resting heart rate and speech from asymptomatic COVID-19 positive individuals. Heart rate and blood oxygen saturation level (SpO_2_) are measured simultaneously at the time of recording the speech using an off-the-shelf pulse oximeter. It should be noted that the pulse rate measured by the pulse oximeter is exactly equal to the heart rate [57]. The total number of speech recordings of healthy individuals at resting heart rate is 84. All the healthy volunteers are in the age group of 25–45 years. Speech samples along with heart rate and SpO_2_ measurements were also obtained from 22 individuals who had tested COVID-19 positive following contact tracing, but with no conspicuous symptoms. The youngest in this category is 32 years and the oldest is 57 years. It should be noted that obtaining speech data of COVID-19 patients was challenging and hence the relatively small set of samples.

The article "Speech as a Biomarker for COVID-19 Detection Using Machine Learning" was published in 2022. Journal: Comput Intell Neurosci.

Speech recording was made using a Logitech headphone equipped with a noise cancellation microphone. While the samples of all the healthy individuals were recorded using the same microphone in the same environment, the speech samples of COVID-19 individuals were recorded with different microphones of the same make and model (Logitech H540) and under different ambient conditions for each. Hence, any variations in speech characteristics arising due to the difference in recording device and ambiance are not taken into consideration. It is reasonable to ignore these variations since the recordings were made in quiet rooms using microphones of the same make and model and therefore have the same technical specifications. Of course, the acoustic effects of the room and background noise, albeit small, are not taken into consideration as it was not possible to bring the COVID-19 patients to the laboratory settings where the recording of healthy individuals was made. Each individual was asked to read the sentence “A quick brown fox jumped over the lazy dogs” which was recorded by turning the microphone “ON”: for 5 seconds. The recording was made in stereo format at a sampling rate of 16000 samples per second (sps) which is the standard sampling rate for wideband representation of speech [58]. The recording is quantized using 2^16^ quantization levels resulting in an audio bit rate of 256 kbps and stored on a computer in uncompressed .WAV format. Heart rate and SpO_2_ level are also concurrently measured at the time of speech recording using a pulse oximeter. The attributes of the data are highlighted in Table 1.

### 2.2. Preprocessing of Speech Data

Unwanted components such as DC bias, which usually gets introduced by PC audio cards [59] and silence intervals due to pauses made by the speaker, are removed by preprocessing each of the speech recordings. DC bias is removed using a 1^st^-order infinite impulse response (IIR) filter, whereas silence intervals are removed by applying a voice activity detection (VAD) mechanism which extracts speech frames containing voice activity. VAD also mitigates noise effects by applying a posteriori signal to noise ratio (SNR) weighting to emphasize reliable segments of voice activity even at low SNR. DC bias removal and VAD are applied as per the implementation provided in [60]. A block diagram of preprocessing steps is shown in Figure 1.

The features of speech that have been used in this study are the short-term Fourier Transform (STFT) coefficients. Features are defined as characteristics of a signal that enables some algorithm to detect an inherent pattern associated with the signal [61]. The premise of detecting COVID-19 from speech features stems from the fact that speech is produced by moving air from the lungs through the vocal cavity. Since there is an interaction between the lungs and heart for the oxygenation of the blood, cardiovascular responses are influenced by activities such as reading and speaking [62]. It is shown in [63] that breathing pattern is affected by the process of speech production. Changes in breathing patterns, in turn, have an effect on the heart rate, and this effect is termed respiratory sinus arrhythmia (RSA) [64]. Several techniques for feature extraction have been proposed in the literature for various applications but predominantly for speaker/speech recognition and speech enhancement. Linear prediction coefficients (LPC), linear prediction cepstral coefficients (LPCC), perceptual linear prediction (PLP), Mel frequency cepstral coefficients (MFCC), Mel frequency discrete wavelet coefficients (MFDWC), feature extraction using principal component analysis (PCA), and wavelets based features are some of the common features that have been reported in the literature [65–70]. STFT represents the time-varying spectral properties of a signal, and for this study, STFT coefficients with a high spectral resolution are used in order to capture subtle differences between closely spaced frequency components. The high spectral resolution is achieved by computing the STFT of long segments of speech, i.e., segment length greater than 500 ms. The high spectral resolution is achieved at the expense of temporal resolution. Since a correlation between physiological parameters and spectral features of speech is evident from existing literature, STFT coefficients with high spectral resolution have been used in this study. The STFT coefficients are used as input features to machine learning algorithms to classify the speech signal as that of COVID-19 positive or not.

The article "Speech as a Biomarker for COVID-19 Detection Using Machine Learning" was published in 2022. Journal: Comput Intell Neurosci.

### 2.3. Statistical Modeling of Speech Features

The most common symptoms of COVID-19 are fever, tiredness, and dry cough, and these may not be conspicuous until about 14 days after getting infected with an average of 5-6 days for the symptoms to become conspicuous. In this article, it is shown using statistical modeling of speech features that it is possible to detect COVID-19 from an individual's speech much before the symptoms become conspicuous so that the person can be quarantined, tested, and provided with medical support at an early stage. At their onset, while symptoms may not be conspicuous to the affected individual or to observers, physiological changes occur in the individual that cause variations in speech characteristics which can be analyzed by artificial intelligence (AI) algorithms. Signal processing and AI can be applied to speech to detect physiological changes which have a direct or indirect relation to one or more of the COVID-19 symptoms. The existence of a correlation between speech characteristics and physiological, psychological, and emotional conditions is well established in the literature. It is therefore possible to detect COVID-19 infection from speech samples of individuals and this possibility is investigated in this article. The relationship between the most common symptoms of COVID-19 and affected physiological parameters is illustrated in Figure 2.

A statistical analysis of speech spectral features is performed by applying maximum likelihood estimation (MLE) to obtain the best statistical distribution along with the distribution parameters that best characterize speech STFT coefficients, statistically. It has been shown in [58] that for speech samples at resting heart rate, STFT coefficients having high spectral resolution are accurately modeled by a Laplacian distribution (LD) with the estimated LD parameters exhibiting small RMS error. The Laplacian distribution is defined as

(1) $$\begin{array}{c} p\left(x\right)=\frac{1}{2b}exp\left(\frac{-\left|x-\mu \right|}{b}\right) \end{array}$$

parameter and *b* > 0 is the scale parameter. The procedure to estimate *μ* and *b*, the RMS error associated with the estimation of *b*, and its lower bound defined as the Cramer-Rao bound (CRB) are provided in [58].

### 2.4. Binary Classification of Speech Samples Using Machine Learning

From the statistical analysis of speech STFT coefficients at the high spectral resolution, it is evident that the RMS error of fitted LD increases as a result of COVID-19 infection. Based on this finding, binary classification of speech signals as COVID-19 positive or COVID-19 negative is investigated by using STFT coefficients as input features to machine learning algorithms. In order to train and develop the AI models, speech samples of healthy as well as COVID-19 positive individuals are used. The trained AI model can then be incorporated into a mobile “app” for early detection of COVID-19, once the desired level of accuracy is achieved and regulatory approvals are obtained. If speech can be used to detect COVID-19, the functionality of the “smartphone” which already has wide proliferation and ubiquitous presence can be extended to alleviate the challenges posed by the pandemic. The results reported in the literature [71–78] are quite promising, providing exciting and interesting answers, giving confidence that research on this topic can lead to the development of mobile applications which can be used not only to detect COVID-19 from human sounds but also for other medical diagnostic/monitoring purposes. COVID-19 diagnosis using only cough recordings is presented in [71]. However, it uses biomarker information such as muscular degradation, vocal cords, sentiment, and lungs/respiratory tract function along with the cough recordings for diagnosis. The relation between COVID-19 symptoms and respiratory system function is highlighted in [72] along with a survey of AI-based COVID-19 diagnoses using human audio signals. Cough and respiratory sounds are used to classify COVID-19 and non-COVID-19 individuals in [73]. Furthermore, it is shown that cough from COVID-19 can be distinguished from healthy individuals' cough as well as cough of asthmatic patients. A project in progress [74] investigates the detection of COVID-19 from human audio sounds using AI. A news feature article in Nature [75] highlights research interest and progress among academic as well as commercial organizations to use the human voice for various diagnostic purposes including COVID-19. AI4COVID-19 is an app that runs an AI algorithm in the cloud to detect COVID-19 from cough sounds and reports promising results, encouraging further collection of labeled cough sounds [76]. An overview of the possibilities, challenges, and use cases of computer audition is presented in [77], which clearly highlights the potential of using sound analysis using AI for COVID-19 diagnosis. A support vector machine (SVM) based method to detect COVID-19 from speech signals is presented in [78] which combines voice signals and symptoms reported by the patient. In contrast to the research available in the literature, this article uses only speech signals without any side information such as symptoms or other biomarker information.

The article "Speech as a Biomarker for COVID-19 Detection Using Machine Learning" was published in 2022. Journal: Comput Intell Neurosci.

The STFT coefficients are labeled as coming from the speech of COVID-19 negative, i.e., healthy (Class 0) and COVID-19 positive (Class 1) individuals. Microsoft Azure Machine Learning Studio (MAMLS) cloud platform is used in this study to perform binary classification, and the performance of classification is analyzed and compared for five state-of-the-art classification algorithms available in MAMLS. Machine learning techniques produce a model for the data by learning the statistical relationship between input data (e.g., STFT coefficients extracted from speech signals) and output data (e.g., class label). The hyperparameters of the produced model are tuned optimally to minimize the classification error in an independent test dataset, resulting in a generalized model that can perform well on the test data set as well. The tuning is performed manually by adjusting the model hyperparameters until the highest value for the “recall” metric is achieved. Good performance on only the training dataset would result in an overfitting solution. A brief description of the five algorithms used for binary classification is provided here for completeness. The block diagram of the methodology used in the work is shown in Figure 3. An overview of the used ML algorithms follows.

Boosted Decision Tree (BDT) is an ensemble learning technique, wherein the succeeding tree corrects the errors of the previous tree to minimize classification error. The complete ensemble of trees is used for correctly predicting the binary class to which the input data belongs [79]. Another classification algorithm based on ensemble learning is the Decision Forest (DF) algorithm, wherein the most popular class is selected depending on the vote from each of the generated trees [80]. Neural Networks (NNs) are a network of interconnected layers of processing units called neurons. A typical NN consists of neurons aggregated into three layers. The first layer is formed by the input feature set which is linked to the output layer via an interconnection of several hidden layers in the middle. Each neuron processes its input variables and its output is passed to the neuron in the subsequent layer [81]. Logistic Regression (LoR) is a statistical technique for analyzing data when a dichotomous outcome is determined by one or more independent variables [82]. Support Vector Machines (SVMs) are based on the principle of recognizing patterns in a multidimensional hyperplane to estimate the maximum margin between samples of binary classes using a multidimensional input feature space [83].

These algorithms have relatively fast training and good performance and are robust to overfitting and have therefore been chosen in this study. The performance of classification models based on each of these algorithms is evaluated using the evaluation metrics listed in Table 2. These evaluation metrics are standard in machine learning literature [84].

The input features used for binary classification are the STFT coefficients of speech from each of the 84 healthy individuals and the 22 COVID-19 positive individuals. Each individual's speech sample comprises 8 segments and STFT coefficients obtained from each speech segment are used as input features for binary classification. As mentioned in Section 4, STFT coefficients are complex numbers; hence, each speech segment comprises “real” and “imaginary” parts of STFT coefficients. The number of frequency points used in the computation of STFT coefficients is 8192, which is obtained as the next power of 2 greater than the segment length. Thus, for each individual speech sample, a matrix of 8192 rows × 8 columns is generated. The real and imaginary parts of the complex STFT coefficients are separated resulting in two separate matrices having dimensions of 8192 rows × 8 columns each. Class label is assigned to each row of these matrices as “Class 0” for healthy individuals' speech samples and “Class 1” for COVID-19 positive individuals. Thus, there are 8192 × 84 = 688,128 rows of STFT coefficients (real part) labeled as Class 0 and 8192 × 22 = 180,224 rows of STFT coefficients (real part) labeled as Class 1. Correspondingly, an equal number of rows are available under each class label containing the “imaginary part” of STFT coefficients.

The article "Speech as a Biomarker for COVID-19 Detection Using Machine Learning" was published in 2022. Journal: Comput Intell Neurosci.

Each row of the real/imaginary part of the STFT coefficients matrix corresponds to a frequency point in the STFT computation, and each column represents a segment of speech. The rows are treated as examples and columns as features since each column of the STFT matrix represents the time-localized spectral features of the speech signals. Every real and imaginary part “x” of STFT coefficients is normalized to lie in the interval [0,1] using a MinMax normalizer as follows:

(2) $$\begin{array}{c} \text{Normalized value}=\frac{x-\text{min}\left(x\right)}{\left[\max\left(x\right)-\text{min}\left(x\right)\right]}. \end{array}$$

Since the statistical distribution for both the real and imaginary parts of speech STFT coefficients is Laplacian, these are treated together without distinction in the context of this work. Thus, the entire dataset comprises 1,736,704 labeled rows, half of which comprise the real part of STFT coefficients and the other half comprise the imaginary part of STFT coefficients, which is saved in .csv format. For binary classification using machine learning, only the rows corresponding to the real part of STFT coefficients are utilized to reduce the time taken for training and cross-validation. The data is split in an 80 : 20 ratio; i.e., 80% of the rows are used for training and the remaining 20% are used for testing. Since the dataset used in this study is highly imbalanced—Class 0 constitutes nearly 80% of the dataset and Class 1 constitutes a little over 20% of the dataset—data splitting is performed with “stratification.” Stratification ensures that each subset of split data has the same class distribution as the entire dataset. The ratio of healthy: COVID-19 + samples in terms of speech recordings is 84 : 22 = 3.8181 : 1. In terms of the STFT coefficients also, this ratio remains the same. Since only the real part of STFT coefficients has been used for binary classification, the ratio healthy: COVID-19 + samples in terms of STFT coefficients is 688128:180224 = 3.8181 : 1. Since stratification has been used, both training and testing data contain STFT coefficients of “healthy” and “COVID+” individuals in the same proportion as 84 :  22 = 3.8181 : 1. Furthermore, the train-test split with stratification at the STFT level ensures permutation of the labeled STFT coefficients across all “individuals”—Class 0 as well as Class 1. Even though the number of speech samples used in this study is small, the number of frequency points (rows) of STFT is large due to the high spectral resolution adopted. The performance evaluation metrics are computed following a 10-fold cross-validation process. Furthermore, as in the data splitting process, stratification is used in the cross-validation process as well to ensure that the class distribution of the training data set is maintained in each fold of cross-validation.

The article "Speech as a Biomarker for COVID-19 Detection Using Machine Learning" was published in 2022. Journal: Comput Intell Neurosci.

## 3. Results

### 3.1. Classification of COVID-19 Samples Based on Statistical Distribution Fitting

LD fitting based on MLE is applied to all the speech samples used in this study—healthy individuals without COVID-19 as well as COVID-19 positive individuals. A comparison of statistical properties of speech STFT coefficients of the two categories of speech samples is performed. The statistical distribution of speech STFT coefficients of healthy individuals, i.e., not infected by COVID-19, is shown in Figure 4 and that of a COVID-19 positive individual is shown in Figure 5.

It is found from Figure 4 that spectral features of the speech of healthy individuals are accurately modeled by LD, with small RMS error as has been established in the literature [58]. In the case of speech samples of COVID-19 positive individuals without any conspicuous symptoms, while the statistical distribution of the STFT coefficients is still closely modeled by LD, the RMS error of the fitted distribution has a nearly 10-fold increase as compared to non-COVID-19 individuals. This increase in the RMS error of the fitted distribution indicates a variation of speech characteristics as a result of COVID-19 infection. The PDFs are obtained by plotting the envelope of histograms of STFT coefficients. The “estimated” PDF represents the fitted distribution based on estimated Laplacian distribution parameters “µ” and “b” and the “actual” PDF is the actual distribution of the STFT coefficients. The Laplacian distribution is therefore a suitable distribution for speech STFT coefficients as the RMS error between the actual and fitted distributions is small.

### 3.2. Performance Evaluation of Binary Classification

The model hyperparameters for each algorithm are tuned and optimized to achieve the best performance in binary classification in terms of the “Recall” metric. The performance evaluation metrics for the five binary classification algorithms used in this study, along with their optimal parameterization, are listed in Table 3. The best performance in terms of precision, recall, accuracy, and F1 score is achieved for the DF algorithm. For the classification application considered in this work, classifying speech spectral features as COVID-19 positive or not, the cost associated with misclassification is very high for “false negative” as compared to “false positive.”

The article "Speech as a Biomarker for COVID-19 Detection Using Machine Learning" was published in 2022. Journal: Comput Intell Neurosci.

Since “recall” provides a measure of correctly predicted positives against the total number of positive examples, it is important for our classification problem to have a high value for this metric. This will minimize misclassifying a COVID-19 positive example as not being COVID-19 positive. While other evaluation metrics have also been determined, “recall” is the more important metric in the context of this work. In Table 3, the values within brackets are the standard deviations of the metrics. Small values for standard deviation indicate that the models are verified with an unbiased dataset which has been achieved by using stratification in the train-test split as well as in cross-validation.

## 4. Discussion

### 4.1. Statistical Distribution of COVID-19 Positive and COVID-19 Negative Speech Samples

The average RMS error for the fitted LD averaged over all the speech samples belonging to each of the two categories is shown in Table 4. This increase in RMS error of the fitted LD in COVID-19 positive samples is attributed to the physiological changes associated with COVID-19 infection which affect the characteristics of speech.

Since the symptoms are not conspicuous among the samples used in this study, the distribution of STFT coefficients of speech is still Laplacian, albeit with a higher RMS error. STFT coefficients being complex numbers, the above findings are valid for both the “real” as well as “imaginary” parts of STFT coefficients and the same has also been shown in [58]. It remains to be seen if the distribution deviates significantly from being Laplacian or even ceases to be Laplacian when the symptoms become more pronounced and conspicuous. The increase in RMS error indicates such a trend. It should be noted that the data used in this study is unbalanced—the dataset from COVID-19 positive individuals is smaller than that of healthy individuals. The results discussed in this section clearly indicate that the statistical properties of speech spectral features are altered as a result of COVID-19 infection. However, as it was not possible to obtain samples of COVID-19 positive individuals whose symptoms are more pronounced and conspicuous, this shall be a subject of future investigation, once such samples are obtained. Due to the prevailing COVID-19 restrictions, access to such individuals has not been possible.

The article "Speech as a Biomarker for COVID-19 Detection Using Machine Learning" was published in 2022. Journal: Comput Intell Neurosci.

### 4.2. COVID-19 Detection on Test Data Using the Binary Classification Models

Finally, the optimally parameterized classification algorithms discussed in Section 2.4 have been tested on the test dataset. As discussed in Section 3.2, the algorithms have been parameterized to optimize the “recall” performance metric. The classification results of 20 samples (rows) from the test data are shown in Table 5 which contains the “actual” and “predicted” classes for the 20 test samples by each of the five classification algorithms. It can be observed from Table 5 that the misclassification of COVID-19 positive as “not positive”, i.e., class 1 being misclassified as Class 0, is the lowest for the DF algorithm. The misclassified values are highlighted in bold and underlined.

For future investigation, concurrently at the time of recording speech samples of individuals, biomedical parameters such as heart rate (pulse oximeter), oxygen saturation (pulse oximeter), blood pressure (digital BP monitor), and temperature (infrared thermometer) have also been measured. These shall be used for future research to develop machine learning-based regression algorithms to predict these biomedical parameters from speech signals. The variations of these parameters among COVID-19 negative and COVID-19 positive individuals shall be analyzed to improve the accuracy of detecting COVID-19 from speech samples. The devices used to measure the biomedical parameters are shown in Figure 6. The e-health sensor platform shown in Figure 6 facilitates direct recording of the biomedical parameter to a PC, thus avoiding the manual entry of data.

A limitation of the work presented in this article is that it cannot distinguish between similar symptoms which may appear due to multiple different causes such as influenza or myocarditis. It requires further research involving speech data from patients with various illnesses that have symptoms similar to COVID-19. This shall be a subject of future work.

## 5. Conclusions

This article investigates the statistical properties of speech spectral features for samples taken from healthy as well as asymptomatic COVID-19 positive individuals. While the statistical distribution for both is Laplacian, the RMS error of the fitted Laplace distribution is higher in the case of asymptomatic COVID-19 positive speech samples. This indicates that spectral properties of speech get altered as a result of physiological changes caused due to COVID-19 infection. It is therefore deduced that there is an associated entropy in speech which can be used to detect COVID-19. STFT coefficients of speech are then used as input features of machine learning-based classification algorithms and the classification performance of five state-of-the-art classification algorithms has been evaluated. All the five classification algorithms exhibit a moderate level of performance having their evaluation metrics values around 70% of their maximum values. The best performance is observed for the DF algorithm which has the highest value for the “recall” metric with a value of 0.7892. “Recall” is the metric used while training the model hyperparameters as a higher recall value means minimizing misclassification of the “false negative” category. The cost of misclassifying a COVID-19 positive sample as a COVID-19 negative is high and hence the choice of recall as the evaluation metric is to be maximized while tuning the model parameters. It is also noted from Table 5 that the misclassification of Class 1 (COVID-19 positive) as Class 0 (COVID-19 negative) is least for the DF algorithm when tested on previously unseen test data. The results obtained are promising and provide evidence that COVID-19 infection can be detected from speech signals of individuals.

The article "Speech as a Biomarker for COVID-19 Detection Using Machine Learning" was published in 2022. Journal: Comput Intell Neurosci.

Speech can be used as a biomedical signal to diagnose various physical and emotional disorders. It can be used to monitor the performance/health conditions of individuals while performing physical activity. The focus of this work, however, is to detect COVID-19 infection by analyzing a person's speech signal. This is possible because speech characteristics of individuals get altered by these conditions as depicted in Figure 7.

The results presented are concurring with similar approaches available in published literature. For example, 100% sensitivity is reported in [71] for asymptomatic cases, but it uses additional biomarker information along with cough sounds. A maximum “recall” value of 0.72 is reported in [73,78] while, in [76], the highest accuracy of 92.85% is reported for binary classification using deep transfer learning.

The results presented in this work can be improved by using a larger dataset comprising different classes of human vocal sounds which should also include samples of individuals of different languages, dialects, and other health conditions. It was intended to collect large datasets by encouraging community participation but that could not be achieved due to regulatory procedures and limitations of funding. Hence, the results presented in this work are based on a small dataset but the findings are encouraging. Future work shall consider using the magnitude of STFT coefficients rather than just the real/imaginary part and also consider the use of other types of audio signal features such as MFCC as input features for ML-based classification. The detection of COVID-19 using speech can facilitate real-time, remote monitoring of infected yet asymptomatic individuals. This will allow early detection of COVID-19 symptoms and help manage the ongoing COVID-19 situation better. It should be noted that the fundamental idea presented in this article is not limited to detecting COVID-19 symptoms only but has broader applications in medical diagnosis and patient monitoring/care. AI can detect changes in human vocal sounds not discernible to the human ear. Smartphone apps that use AI algorithms to analyze human vocal sounds for diagnosis, screening, and monitoring can be extremely useful and are expected to play a vital role in future healthcare technologies.

The article "Speech as a Biomarker for COVID-19 Detection Using Machine Learning" was published in 2022. Journal: Comput Intell Neurosci.

## Figures and Tables

**Figure 1:** Speech preprocessing.

**Figure 2:** Biological parameters correlated to speech and COVID-19 symptoms.

**Figure 3:** Block diagram of the methodology used.

**Figure 4:** Statistical properties of speech STFT coefficients of a healthy person (without COVID-19).

**Figure 5:** Statistical properties of speech STFT coefficients of an infected person (with COVID-19).

**Figure 6:** Devices used for measuring biomedical parameters along with speech for future analysis.

**Figure 7:** Possible applications of the proposed research.

**Table 1:** Attributes of data used in this study.

	Age group (years)	No. of recordings	Sampling rate (sps)	Quantization depth (bits)	Audio bit rate (kbps)	Audio format	Other parameters measured
Healthy	25–45	84	16000	16	256	.wav	Heart rate, SpO_2_
COVID+	32–57	22					

**Table 2:** Evaluation metrics for binary classification.

Evaluation metric	Definition	Notations
Binary classification		
Precision (PRE)	PRE = *t*_*p*_/*t*_*p*_+ *f*_*p*_	tp–Total no. of true positive samples
Recall (REC)	REC = *t*_*p*_/*t*_*p*_+ *f*_*n*_	tn–Total no. of true negative samples
Accuracy (ACC)	ACC = *t*_*p*_+ *t*_*n*_/*t*_*p*_ + *t*_*n*_+ *f*_*p*_ + *f*_*n*_	fp–Total no. of false positive samples
F1-score	*F*1=2*∗P*_*RE*_*∗R*_*EC*_/*P*_*RE*_+*R*_*EC*_	fn – Total no. of false negative samples
Area under RoC curve	(AUC) AUC =∫_0_^1^RoC	RoC - receiver operating characteristic curve

**Table 3:** Performance metrics for binary classification algorithms.

Classification algorithms	Optimal Parameterization	Performance metrics Mean value (standard deviation)				
		A_CC_	P_RE_	R_EC_	F1 score	AUC
BDT	No. of Leaves: 16 Learning rate: 0.05 No. of trees: 100	0.724 (0.048)	0.714 (0.037)	0.7037 (0.063)	0.7088 (0.052)	0.717 (0.053)
DF	Random split Count: 128 Maximum Depth: 32 No. of decision trees: 16	0.7317 (0.021)	0.7421 (0.017)	0.7892 (0.081)	0.7649 (0.025)	0.755 (0.017)
NN	Learning rate: 0.001 No. of hidden Nodes: 314	0.711 (0.031)	0.7271 (0.043)	0.7188 (0.018)	0.7229 (0.029)	0.7616 (0.095)
LoR	Optimization Tolerance: 1e-06 L1 regularization weight: 1 Memory size for L-BFGS: 18	0.6741 (0.019)	0.6805 (0.024)	0.6161 (0.027)	0.6467 (0.019)	0.6874 (0.065)
SVM	Lambda – 0.001	0.694 (0.017)	0.673 (0.074)	0.6027 (0.019)	0.6359 (0.011)	0.6619 (0.037)

The article "Speech as a Biomarker for COVID-19 Detection Using Machine Learning" was published in 2022. Journal: Comput Intell Neurosci.

**Table 4:** Average RMS error of the fitted LD distributions.

Category	Average RMS error of fitted LD
Without COVID-19	0.00354
With COVID-19	0.01271

**Table 5:** Test evaluation for binary classification

Test sample	Actual class	Predicted class				
		BDT	DF	NN	LoR	SVM
1	0	0	1	0	0	1
2	1	1	1	**0**	1	1
3	1	1	1	1	**0**	**0**
4	0	1	0	1	1	1
5	1	1	1	**0**	1	1
6	0	0	0	0	0	0
7	1	**0**	**0**	1	1	1
8	1	1	1	1	**0**	**0**
9	1	**0**	**0**	**0**	1	1
10	0	1	0	0	1	1
11	1	**0**	1	1	1	1
12	0	0	1	1	0	0
13	0	1	0	1	1	0
14	1	1	1	1	**0**	1
15	0	0	0	0	0	1
16	0	1	1	0	0	1
17	1	1	1	**0**	**0**	**0**
18	1	**0**	1	1	1	1
19	0	0	0	1	0	1
20	1	1	1	1	0	1

## Data Availability

The speech recordings and the features data used to support the findings of this study have not been made available because the participants have not consented to their data being shared with any third party.
